The article "Mental Health Problems Among Front-Line Healthcare Workers Caring for COVID-19 Patients in Vietnam: A Mixed Methods Study" was retracted in 2024. Reasons: duplicate publication; overlap with earlier publications.

# Mental Health Problems Among Front-Line Healthcare Workers Caring for COVID-19 Patients in Vietnam: A Mixed Methods Study

**DOI:** 10.3389/fpsyg.2022.858677

**Published:** 2022-04-15

**Authors:** Thu Kim Nguyen, Ngoc Kim Tran, Thuy Thanh Bui, Len Thi Tran, Nhi Tho Tran, Mai Tuyet Do, Tam Thanh Nguyen, Huong Thi Thanh Tran

**Affiliations:** ^1^Hanoi Medical University, Hanoi, Vietnam; ^2^National Institute of Hygiene and Epidemiology, Hanoi, Vietnam; ^3^National Hospital of Obstetrics and Gynecology, Hanoi, Vietnam; ^4^Vietnam National Cancer Hospital, Hanoi, Vietnam; ^5^BasicNeeds Vietnam, Hanoi, Vietnam

**Keywords:** mental health problems, front-line, healthcare workers, COVID-19, Vietnam, mixed methods

## Abstract

**Aim:**

Healthcare workers have directly provided care for COVID-19 patients, and have faced many additional sources leading to poor mental health. The study aimed to investigate the mental health problems and related factors among healthcare staff in Vietnam.

**Methods:**

A descriptive cross-sectional mixed methods study, combining quantitative and qualitative research methods, was performed among 400 healthcare workers working at the National Hospital for Tropical Diseases and Ninh Binh General Hospital from the first day of treatment for COVID-19 patients to May 01, 2020.

**Results:**

The results showed that 8.0% of participants had stress, 17.5% of participants had anxiety, and 14.8% of participants had depression. Approximately 50% of participants reported that they had at least one of these symptoms. The findings illustrated that stress, anxiety, and depression were associated with the position in a hospital, health status during the COVID-19 pandemic, family members/relatives infected with COVID-19, physical and mental support from friends, family, and community, department, years of working, and the average work hours per day of healthcare workers exposed to COVID-19.

**Conclusion:**

During the COVID-19 pandemic, healthcare workers who worked in the hospital providing treatment and care for COVID-19 patients dealt with mental health problems such as stress, anxiety, and depression. It is necessary to promote mental health among healthcare workers, to contribute to the fight against the COVID-19 outbreak in Vietnam.

## Introduction

In recent years, coronavirus disease (COVID-19) has been the biggest pandemic worldwide due to its speed and scale of transmission (Verity et al., 2020). The first known cases were reported in Wuhan, China in December 2019 before spreading rapidly around the world (Verity et al., 2020; Zhu et al., 2020a). After that, the World Health Organization (WHO) declared the novel coronavirus outbreak a worldwide pandemic in March 2020 (Cucinotta and Vanelli, 2020). As of May 30, 2020, the number of cases and deaths globally due to COVID-19 was reported as 6,029,950 and 366,802, respectively (General Department of Preventive Medicince, 2020). In Vietnam, the first cases, two Chinese people in Ho Chi Minh city, were identified in January 2020 (General Department of Preventive Medicince, 2020). The Vietnam government has immediately decided to suspend the entry of all foreigners since March 22^nd^, 2020 (Le et al., 2021). Vietnam is an example of one of the best-organized epidemic control programs worldwide due to the rapid response, a decisive central government, and a proactive containment strategy (Le et al., 2021).

As with all communicable diseases, the COVID-19 outbreak has affected all individuals and communities in terms of their health (Cincidda et al., 2021; Ongaro et al., 2021), particularly healthcare workers who have engaged in the fight against COVID-19. They are at higher risk of COVID-19 infection as well as psychological distress and symptoms of mental health problems when coping with the COVID-19 pandemic (Chew et al., 2020). Few studies were performed to determine several risk factors associated with the mental health of healthcare workers, including symptoms of stress, anxiety, and depression during the COVID-19 pandemic (Pappa et al., 2020). In a study conducted in China, the results illustrated that 50.4% of healthcare workers suffered stress, and 44.6% of those coped with anxiety in the COVID-19 pandemic (Lai et al., 2020). Further, other factors in terms of the demanding nature of their work, such as long working hours, risk of infection, shortages of protective equipment, loneliness, physical fatigue, and separation from families were associated with the increase in adverse mental health outcomes among these subjects (Kang et al., 2020).

Until May 2020, there were few COVID-19 patients treated, with 270 cases and no deaths in Vietnam (General Department of Preventive Medicince, 2020). The study was conducted in two hospitals in the north region: the National Hospital for Tropical Diseases in Hanoi and Ninh Binh General Hospital, because they were largest among the few hospitals approved to provide treatment for COVID-19 patients by the Vietnam Ministry of Health (MOH). Healthcare staff in these hospitals contributing to treatment for COVID-19 patients had to deal with the high risk of COVID-19 infection and its damaging impact on their health, in particular on mental health (Lai et al., 2020; Rajkumar, 2020). To our knowledge, this is the first study in Vietnam to explore the relationship between potential risk factors and mental health among healthcare workers during the COVID-19 outbreak. To provide support solutions enhancing and maintaining mental well-being, this study aimed to examine mental health issues such as stress, anxiety, and depression, and determine potential factors associated with mental health among healthcare staff in Vietnam.

## Materials and Methods

### Study Design and Participants

A descriptive cross-sectional mixed methods study, combining quantitative and qualitative research methods, was conducted in two separate hospitals having treatment for COVID-19 patients in the Northern region of Vietnam, including the National Hospital for Tropical Diseases in Hanoi and Ninh Binh General Hospital, from May1, 2020, to August 30, 2020. The evaluation period for this study was from the date of two hospitals starting the treatment for COVID-19 patients to May 1, 2020.

In the quantitative study, subjects were recruited following several inclusion criteria: (1) healthcare staff working in hospitals engaged in the treatment of COVID-19 patients; (2) worked during the evaluation period (from the first day that two hospitals started the treatment of COVID-19 patients to May 1st, 2020); and (3) agreed to participate in this study. The exclusion criteria was that they did not agree to take part in the study. After applying purposive sampling, the total sample size was estimated at 400 healthcare staff, including 260 and 140 individuals working in the National Hospital of Tropical Diseases and Ninh Binh General Hospital, respectively. 100% of interviewed subjects agreed to participate in the study.

In a qualitative study, a structured interview was conducted with 15 healthcare workers in two hospitals, including 10 persons in National Hospital for Tropical Diseases and 5 individuals in Ninh Binh General Hospital. Among those, participants were selected as following:

- 3 doctors directly treated COVID-19 patients.
- 6 nurses directly cared for COVID-19 patients.
- 3 other positions were exposed to COVID-19 (especifically, the hospital orderly employee is the person who directly assist the nurses to take care of patients in clinical departments).
- 3 doctors or nurses had no direct contact with COVID-19 patients.

### Data Collection and Measurement

The mixed method design was used to address the main objects, in which qualitative and quantitative data was collected simultaneously, analyzed independently, then combined to inform the interpretation.

#### Quantitative Questionnaire-Based Study

We used a structured self-report questionnaire to collect the data. All eligible subjects were invited to participate in the study. The questionnaire provided to participants consisted of two major components: (1) Socioeconomic characteristics, (2) Depression Anxiety Stress Scale (DASS-21).

##### Socioeconomic Characteristics of Participants

All healthcare staff was asked several questions about their personal information, including demographic characteristics, potential factors, and mental health problems.

##### Depression Anxiety Stress Scale (DASS-21)

The DASS-21 scale is a quantitative measure of distress (depression, anxiety, and stress) constructed from the psychometric characteristics of the 21-item version that is validated in Vietnam (Tran et al., 2013). Each item ranges on a 4-point Likert scale, consisting of 0 “Did not apply to me at all,” 1 “Applied to me to some degree or some of the time,” 2 “Applied to me to a considerable degree or a good part of the time,” and 3 “Applied to me very much, or most of the time.” The scores for Depression, Anxiety and Stress are calculated by adding the scores of the sub-categories, then multiply by 2. In which, depression is classified according to 5 levels including normal (0–9), mild (10-) 13), moderate (14–20), severe (21–27), very severe (28 and more). Anxiety is classified according to 5 levels including normal (0–7), mild (8–9), moderate (10–14), severe (15–19), very severe (20 and more). Stress is classified into 5 levels including normal (0–14), mild (15–18), moderate (19–25), severe (26–33), very severe (34 and more).

#### Qualitative Interview Study

A structured interview was designed as a list of predetermined questions to supplement the explanation for the quantitative study: (1) to investigate subjects’ mental experiences and symptoms of stress, anxiety, and depression while treating and caring for COVID-19 patients, (2) to explore related factors from the detailed insights of individual, family/society and work environment. The interviews were conducted by two researchers who were trained in conducting qualitative interviews and has expertise in psychology. Each interview involved one interviewee at the time and took 50–60 min per person. The interviewer asked open-ended questions and let the subject describe their own experience and feelings. Participant who agreed to participate had to complete the consent form before continuing to the survey questions. The survey was kept confidential and anonymous, and the participants could terminate their participation at any time.

### Data Analysis and Statistical Methods

To address the main aims of the study, both descriptive and analytical statistics for quantitative data were analyzed by utilizing STATA version 12.0. Qualitative variables were presented as frequency and percentage (%), while quantitative variables were presented as mean and standard deviation (SD). Odd ratios (OR) were used to determine factors associated with the average score of the measurement scale for stress, anxiety, and depression. A value of p (p) of 0.05 was considered statistically significant. For the qualitative study, data was entered and arranged in Microsoft Excel.

### Ethical Consideration

The study protocol, materials, and procedures were approved by the Institutional Review Board at Dinh Tien Hoang Institute of Medicine (IRB-VN02010-10/2015). All subjects were provided with the sufficient information regarding the study before they signed the informed consent form.

## Results

Table 1 shows the demographic characteristics of 400 participants in two hospitals having the biggest total number of COVID-19 patients in the northern region of Vietnam. 60% of healthcare staff worked at the National Hospital for Tropical Diseases in Hanoi (240 individuals). The majority of respondents were female (63%) and aged 35 or under (79%).

**Table 1:** Characteristics of participants.

Characteristics	Ninh Binh general hospital		National hospital for tropical diseases		Total		Value of *p*
	*n*	%	*n*	%	*n*	%	
Total	140	40.0	260	60.0	400	100.0	
*Gender*							
Male	53	37.9	95	36.5	148	37.0	0.79
Female	87	62.1	165	63.5	252	63.0	
*Age*							
<=35	123	87.9	193	74.2	316	79.0	<0.01
>35	17	12.1	67	25.8	84	21.0	
*Marital status*							
Single	58	41.4	90	34.6	148	37.0	0.42
Married	80	57.2	167	64.2	247	61.8	
Divorce	1	0.7	2	0.8	3	0.8	
Widow	1	0.7	1	0.4	2	0.4	
*Education*							
Postgraduate	19	13.6	60	23.1	79	19.8	<0.01
University	65	46.4	90	34.5	155	38.7	
College	37	25.4	94	36.1	131	32.7	
Others	19	13.6	16	6.2	35	8.8	
*Position in hospital*							
Doctor	22	15.7	87	33.5	109	27.3	<0.01
Nurse	82	58.6	109	41.9	191	47.7	
Hospital orderly	–		4	1.5	4	1.0	
Others	36	25.7	60	23.1	96	24.0	
*Monthly income*							
= 5 million VND ($220)	112	80.0	224	86.2	336	84.0	0.11
< 5 million VND ($220)	28	20.0	36	13.8	64	16.6	

“–“ dash: no cases was reported.

Table 2 represents that the percentage of anxiety (17.5%) among healthcare staff was higher than the proportions of stress and depression (8 and 14.8%, respectively). The rate of stress was lower in the National Hospital for Tropical Diseases than that in Ninh Binh General Hospital, whereas the rates of anxiety and depression were higher in the National hospital for Tropical Diseases were lower than those in Ninh Binh General Hospital. However, these differences between two hospitals were not statistically significant. The percentage of anxiety among health care staff was higher than the proportion of stress and depression. In Figure 1, the percentages of mild level of depression and stress were higher than the proportions of other levels (7.5 and 4.7%, respectively), followed by moderate level of these problems (6.0 and 1.8%, respectively). For anxiety, the proportion of moderate level was the highest at 10.0%, followed by mild level with 4.0%.

**Table 2:** Stress, anxiety, and depression among healthcare workers in Vietnam.

Mental health	Ninh Binh general hospital		National hospital for tropical diseases		Total		Value of *p*
	*n*	%	*n*	%	*n*	%	
Stress	15	10.7	17	6.5	32	8.0	0.43
Anxiety	20	14.3	50	19.2	70	17.5	0.21
Depression	18	12.9	41	15.8	59	14.8	0.14

**Figure 1:** The level of stress, anxiety, and depression among healthcare workers in Vietnam.

The qualitative study revealed some common reasons that can caused the healthcare workers’ stress, anxiety, and depression during the working time on the COVID-19 outbreak, especially the lack of knowledge about COVID-19 disease and its transmission can cause anxiety.

*“Firstly, this is a new disease, and I have no idea about it. Secondly, I do not know its transmission. So, I am extremely worried”* (Mr. TA, 54 years old).

Furthermore, hearing the information that other colleagues were infected with COVID-19 made the healthcare worker suffer more stress, anxiety, and depression, particularly while working at a high risk of COVID-19 infection.

*“At that time, case number 17 caused a huge community infection, so when I heard the news that there was a new case, I was afraid, afraid of getting infected because in the world, several medical workers were infected, some died. Thus, when I contact patients, I am very scared”* (Mrs. L, 32 years).

*“Front-line healthcare workers have suffered stress and anxiety, but others who do not directly provide care for patients are normal …”* (Mrs. H, 30 years).

Other reason of psychological problems among participants was the lack of belief in personal protective equipment (PPE).

*“There are over 10 cases of positive hospitalization per day that makes me feel worried because I am scared of being infected, even though I have had PPE but I am still at a higher risk than others. Taking off PPE is more scary than puting it on, because wearing PPE many hours causes one to sweat profusely. Usually it is all a muck of sweat, I am just scared about PPE, I mean, the risk of splashing or spraying specimens on skin. It is extremely dangerous. Everyone is worried about that”* (Mrs. Th).

Not only the concern of personal health, the health care workers also got stressed because of family issues. In the quarantine place, healthcare staff are more worried about their family members, particularly their parents and childrens’ health.

*“I am worried that my grandmother is living by herself, and I can not take care of my child. I am afraid of unexpected accidents”* (Mrs. H, 31 years).

*“My child, my husband, and I have to go for several months so I worry and think a lot” (Mrs. Th).*

Table 3 shows several factors that might affect the mental health of healthcare workers. Odd ratios were calculated to determine the relationship between associated factors and mental health issues among healthcare staff (Table 4). Several variables were included in the model, including gender, position in a hospital, health status during COVID-19, family members or friends infected with COVID-19, physical and mental support from friends, family, and community, department, experience year, the average working time during COVID-19, and direct contact with COVID-19 patients. The results illustrated that being a doctor (OR = 3.83; 95% CI: 1.05–14.03), having bad or normal health during COVID-19 (OR = 3.18; 95%CI: 1.51–6.69), having family members/friends infected with COVID-19 (OR = 6.50; 95%CI: 2.70–15.70), having over 5-year experience (OR = 0.34; 95% CI: 0.12–0.90), their average work hours over 8 h during COVID (OR = 3.60; 95%CI: 1.43–9.05), statistically significantly associated with the development of stress.

**Table 3:** Reported feelings of stress, anxiety and depression among healthcare workers in Vietnam.

Variables	Stress		Anxiety		Depression	
	Yes	No	Yes	No	Yes	No
	*n* (%)	*n* (%)	*n* (%)	*n* (%)	*n* (%)	*n* (%)
Total	32	368	70	330	59	341
*Gender*						
Male	13 (40.6)	135 (36.7)	24 (34.3)	124 (37.6)	23 (39.0)	125 (36.7)
Female	19 (59.4)	233 (63.3)	46 (65.7)	206 (62.4)	36 (61.0)	216 (63.3)
*Position in hospital*						
Doctors	12 (37.5)	97 (26.4)	23 (32.9)	86 (26.1)	25 (42.4)	84 (24.6)
Nurse	17 (53.1)	174 (47.3)	40 (57.1)	151 (45.8)	30 (50.8)	161 (47.2)
Orderly	0 (0)	4 (1.1)	0 (0)	4 (1.2)	4 (6.8)	0 (0)
Others	3 (9.4)	93 (25.3)	7 (10.0)	89 (27.0)	4 (6.8)	92 (27.0)
*Health status during COVID-19*						
Very good/good	16 (50.0)	280 (76.1)	35 (50.0)	261 (79.1)	33 (55.9)	263 (77.1)
Normal/bad	16 (50.0)	15 (4.1)	35 (50.0)	69 (20.9)	26 (44.1)	78 (22.9)
*Family member/friend infected with COVID-19*						
No	22 (68.8)	343 (93.2)	56 (80.0)	309 (93.6)	46 (78.0)	319 (93.5)
Yes	10 (31.3)	24 (6.5)	14 (20.0)	20 (6.1)	13 (22.0)	21 (6.2)
*Physical and mental support from friends, family, and community*						
Yes	30 (93.8)	330 (89.7)	61 (87.1)	299 (90.6)	48 (81.4)	312 (91.5)
No	2 (6.3)	38 (10.3)	9 (12.9)	31 (9.4)	11 (18.6)	29 (8.5)
*Department*						
Emergency	5 (15.6)	84 (22.8)	15 (21.4)	74 (22.4)	14 (23.7)	75 (22.0)
Treatment	22 (68.8)	159 (43.2)	43 (61.4)	138 (41.8)	38 (64.4)	143 (41.9)
Para clinical	1 (3.1)	55 (14.9)	8 (11.4)	48 (14.5)	4 (6.8)	52 (15.2)
Others	4 (12.5)	70 (19.0)	4 (5.7)	70 (21.2)	3 (5.1)	71 (20.8)
*Experience year*						
≤5 years	27 (84.4)	238 (64.7)	48 (68.6)	217 (65.8)	42 (71.2)	223 (65.4)
>5 years	5 (15.6)	130 (35.3)	22 (31.4)	113 (34.2)	17 (28.8)	118 (34.6)
*The average working time during COVID-19*						
≤8 h/day	6 (18.8)	167 (45.4)	27 (38.6)	146 (44.2)	15 (25.4)	158 (46.3)
>8 h/day	26 (81.3)	201 (54.6)	43 (61.4)	184 (55.8)	44 (74.6)	183 (53.7)
*Direct contact with COVID-19 patients*						
Yes	13 (40.6)	182 (49.5)	40 (57.1)	155 (47.0)	35 (59.3)	160 (46.9)
No	19 (59.4)	186 (50.5)	30 (42.9)	175 (53.0)	24 (40.7)	181 (53.1)

**Table 4:** Association between potential factors and stress, anxiety, and depression among healthcare workers in Vietnam.

Variables	Stress OR (95% CI)	Anxiety OR (95% CI)	Depression OR (95% CI)
*Gender*			
Female	1	1	1
Male	1.18 (0.56–2.45)	0.87 (0.50–1.49)	1.11 (0.62–1.95)
*Position in hospital*			
Others	1	1	1
Doctor	3.83 (1.05–14.03)	3.40 (1.39–8.33)	6.85 (2.28–20.48)
Nurse	3.03 (0.86–10,60)	3.37 (1.45–7.84)	4.29 (1.46–12.55)
*Health status during COVID-19*			
Very good/good	1	1	1
Normal/bad	3.18 (1.51–6.69)	3.78 (2.17–6.60)	2.66 (1.48–4.75)
*Family member/friend infected with COVID-19*			
No	1	1	1
Yes	6.50 (2.70–15.70)	3.90 (1.80–8.20)	4.30 (2.00–9.30)
*Physical and mental support from friends, family, and community*			
Yes	1	1	1
No	0.60 (0.10–2.50)	1.40 (0.60–3.10)	2.50 (1.10–5.30)
*Department*			
Others	1	1	1
Emergency	1.04 (0.27–4.03)	3.55 (1.12–11.21)	4.42 (1.22–16.02)
Treatment	2.42 (0.80–7.29)	5.45 (1.88–15.81)	6.29 (1.88–21.08)
Para clinical	0.32 (0.03–2.93)	2.92 (0.83–10.23)	1.82 (0.39–8.48)
*Experience year*			
≤5 years	1	1	1
>5 years	0.34 (0.12–0.90)	0.88 (0.51–1.53)	0.70 (0.42–1.40)
*The average working time during COVID-19*			
≤8 h per day	1	1	1
>8 h per day	3.60 (1.43–9.05)	1.26 (0.74–2.15)	2.53 (1.35–4.76)
*Direct contact with COVID-19 patients*			
Yes	1	1	1
No	0.70 (0.33–1.46)	1.50 (0.89–2.54)	1.65 (0.93–2.90)

Moreover, being a doctor (OR = 3.40; 95% CI: 1.39–8.33 and OR = 6.85; 95% CI: 2.28–20.48, respectively), being a nurse (OR = 3.37; 95% CI: 1.45–7.84 and OR = 4.29; 95% CI: 1.46–12.55, respectively), having bad or normal health during COVID-19 (OR = 3.78; 95% CI: 2.17–6.60 and OR = 2.66; 95% CI: 1.48–4.75, respectively), having family members/friends infected with COVID-19 (OR = 3.90; 95% CI: 1.80–8.20 and OR = 4.30; 95% CI: 2.00–9.30, respectively), having no physical and mental support from friends, family and community (OR = 2.50; 95% CI: 1.10–5.30), working in the emergency department (OR = 3.55, 95% CI: 1.12–11.21 and OR = 4.42; 95% CI: 1.22–16.02, respectively), working in the treatment department (OR = 5.45; 95% CI: 1.88–15.81 and OR = 6.29; 95% CI: 1.88–21.08, respectively), their average work hour over 8 h during COVID-19 (OR = 2.53; 95% CI: 1.35–4.76) were also significantly related to development of anxiety and depression.

In particular, some healthcare staff confessed that sometimes they felt pressured because they had no preparation for receiving patients with COVID-19.

*“People in our department have not determined to provide care for COVID-19 patients before we were informed that the department would receive patients on the next day. No one has been mentally prepared, so we are nervous …”* (Nurse, Mrs. Th, 32 years).

They also got stress, anxiety, and depression even though they were thoroughly trained because the clinical practice was totally different from the theories.

*“The theory taught was completely different from the practical reality, some individuals were embarrassed …”* (Doctor, Mr. Th, 54 years).

Despite the fact that medical workers experienced mental health issues during the COVID-19 pandemic, the encouragement and support of friends, family, and the community helped them to reduce their stress, anxiety, and depression.

*“The happiness when returning home is multiplied, I receive a warm welcome from my family and others”* (Nurse, Mrs. Th, 32 years old).

*“My friends heard the news and called me to ask that they had a desire to support masks and other supplements”* (Doctor, Mr. Th, 54 years old).

However, they always maintain a high level of obligation and responsibility to their work, patients, and community.

*“During the COVID-19 pandemic, we were here 24 h per day. We did not go out of the quarantine place”* (Doctor, Mr. Th, 54 years old).

*“We have four shifts per day, six hours per shift. We work a six-hour shift per day. In cases in which the health condition of a patient becomes severe, we had to work more than a shift per day. We had to do everything, such as receiving patients, providing clothes, putting off their clothes, and providing infusion. I had to do it on my own because no family members of patients were allowed to come in …”* (Nurse, Mrs. L, 32 years old).

## Discussion

As an aspect of the fight against the COVID-19 outbreak, healthcare workers are more likely to suffer adverse mental health outcomes when they have the closest contact with COVID-19 patients. Anxiety was a prevalent mental problem among medical staff. The frequent stress-related symptoms were tiredness (31.0%), insomnia (29.5%), inappetence (27.5%), and headache (22.8%).

Vietnam has rapidly responded and succeeded in controlling the spread of COVID-19 during the early period of the outbreak (Ha et al., 2020; Le et al., 2021). Since the COVID-19 pandemic was declared by WHO, the Vietnam government immediately enacted the appropriate policies and implemented drastic measures, including suspending entry for all foreigners and imposing a strict quarantine period (Ha et al., 2020). Further, the efforts of the health system such as the provincial Center for Diseases Control (CDC) network, hospitals as well as healthcare workers in the control, prevention, and curative care of COVID-19 have also played an important role in the effective measures (Ha et al., 2020). The reasonable decision to eliminate the wide spread of the COVID-19 outbreak in Vietnam might support reducing the level of psychological problems and the burden of healthcare staff in providing treatment and care for COVID-19 patients (Ha et al., 2020).

The COVID-19 pandemic has caused psychological problems in medical staff (Ho et al., 2020). Frontline healthcare workers have faced the poor health status of COVID-19 patients as well as patients’ deaths (Vizheh et al., 2020). Further, the fear of being infected, isolation from their family, and the pressure of workload may be associated with many symptoms of psychological disorders (Vizheh et al., 2020). Similar to other nations worldwide, healthcare staff in Vietnam were under pressure due to coping with the new infectious disease, COVID-19, and were in dire need of mental health support. Rates of stress and anxiety in our study were lower than those figures in China (29.8 and 24.1%, respectively; Zhu et al., 2020b) and another study in Spain (63.0 and 67.6%, respectively; Odriozola-González et al., 2020). The rate of depression in our study was higher than that in China (12.1%; Zhu et al., 2020b), but was lower than that in Spain (55.9%; Odriozola-González et al., 2020). The rates of anxiety and depression were lower in our study than those in a study performed in the United States (33 and 21%, respectively; Hassamal et al., 2021). The reason why the rates of mental health problems among Vietnamese medical staff were lower than those in other nations might be due to the COVID-19 incidence and mortality rates in Vietnam were lower than those in many countries (World Health Organization). Compared to the rates of problems in mental well-being during other infectious diseases such as the severe acute respiratory syndrome (SAR) and the Middle East Respiratory Syndrome (MER) outbreaks, the rates of stress, anxiety and depression among healthcare workers were greater than our results. It might be explained that the fatality rate of SARS-CoV-2 was low compared to SARS and MERS (Vizheh et al., 2020). Healthcare staff in Vietnam were more likely to experience mild levels of depression and stress, and a moderate degree of anxiety. Compared to the results of the other study, the majority of medical staff in China (36.5%) coped with a mild degree of depression and anxiety (Lai et al., 2020). The consequences might be understandable due to the fear of increasing infections for themselves and their loved ones (Ho et al., 2020). Further, they had several symptoms similar to those of COVID-19 that might have been caused by the overwork (Ho et al., 2020).

The results showed that, compared with those who had very good or good health during the COVID-19 outbreak, medical staff members who had bad or normal health status reported more stress, anxiety, and depression. Additionally, there was a significant association between suffering stress, anxiety, and depression and having loved ones or friends infected with COVID-19 among healthcare workers. They tried to balance their responsibilities with their patients as well as the fear of transmitting it to their family members (Johnson et al., 2021). Besides, doctor in hospitals seems to experience more stress, anxiety, and depression. This finding differed the results in a study of Spain in which being doctor only significantly related to anxiety (Luceño-Moreno et al., 2020).

In addition, medical staff having over 5-year of experience reported less stress when participating in the fight against the COVID-19 pandemic. In another study in the United States, medical staff with 6-to-9-year of working experience were two times more likely to face moderate or severe depression compared to those with 10 or more years of work experience (Hassamal et al., 2021). Another study in China demonstrated that working over 10 years was related to stress, anxiety, and depression (Zhu et al., 2020b). However, working over 8 h was significantly associated with an increase in stress and depression. Shorter working hours should be considered to reduce the pressure on their careers and improve their mental well-being (Ho et al., 2020; Kang et al., 2020). Another finding was that healthcare workers who worked as nurse positions were more likely to experience anxiety and depression, which was similar to the result of a study in China (Lai et al., 2020). Moreover, our study reported that healthcare workers working in the emergency and treatment departments were significantly associated with an increase in anxiety and depression. A study conducted in Saudi Arabia indicated that medical staff who provided treatment for COVID-19 patients were at high risk of psychological problems, including stress, anxiety, and depression (Al-Mansour et al., 2021).

On the other hand, these findings indicated that having belief in PPE and direct engagement with COVID-19 patients was not significantly associated to stress, anxiety and depression among healthcare staff in Vietnam. The results in our study differed from those in China in which healthcare workers having direct contact with COVID-19 patients were more likely to suffer stress, anxiety, and depression (Lai et al., 2020). Mental health supports, including colleagues and supervisors and clear communication of directives and precautionary measures, might reduce psychological symptoms (Al-Mansour et al., 2021). In Saudi Arabia, a study illustrated that there was a negative correlation between social support and stress (Al-Mansour et al., 2021). Healthcare workers who lacked the emotional support from family and society were more likely to experience stress compared to others (Arafa et al., 2021). It is necessary to provide adequate training on infection control and the mental health support services for frontline medical staff (Ho et al., 2020). Nevertheless, psychological services have not been considered to enhance the mental health of healthcare workers in Vietnam.

In our study, there were several limitations. Firstly, the study was conducted before the second wave of the COVID-19 pandemic occurred in Vietnam, and the incidence and mortality due to COVID-19 was low. That might have led to the low rates of mental health problems among healthcare workers in two separate hospitals. Secondly, the median age of participants is low less than 35 years old, because the majority of healthcare workers participating in the fight with COVID-19 pandemic were young. The psychological problems of young employees may be different from those of older employees, so the representativeness of the study sample is limited. Additionally, the other limitation was the small sample size, and that healthcare workers participating in the study were in the north region, which might not represent the general healthcare staff in Vietnam. Further studies should be performed with a greater sample size and more hospitals in all regions of Vietnam.

## Conclusion

During the COVID-19 pandemic, healthcare workers who worked in the hospital providing treatment and care for COVID-19 patients deal with the mental health problems such as stress, anxiety and, depression with several symptoms. This study implies that promoting mental health for healthcare workers should be considered as an important component of the prevention and control programs in the fight against the COVID-19 outbreak in Vietnam. Further studies should be implemented to examine the adequate supports provided to healthcare workers to enhance their mental well-being.

## Data Availability Statement

The raw data supporting the conclusions of this article will be made available by the authors, without undue reservation.

## Ethics Statement

The studies involving human participants were reviewed and approved by the study protocol, materials, and procedures were approved by the Institutional Review Board at Dinh Tien Hoang Institute of Medicine, Hanoi, Vietnam (No. IRB-VN02010-10/2015). The patients/participants provided their written informed consent to participate in this study.

## Author Contributions

TKN, NKT, and HT designed the study. TKN, TB, and LT collected the data. TKN, NKT, and NTT analyzed the data. TKN, MD, and HT interpreted the data and drafted the manuscript. TKN, TTN, and HT reviewed the data analysis and manuscript. All authors approved the final version for publication.

## Conflict of Interest

The authors declare that the research was conducted in the absence of any commercial or financial relationships that could be construed as a potential conflict of interest.

## Publisher’s Note

All claims expressed in this article are solely those of the authors and do not necessarily represent those of their affiliated organizations, or those of the publisher, the editors and the reviewers. Any product that may be evaluated in this article, or claim that may be made by its manufacturer, is not guaranteed or endorsed by the publisher.
